# How to Improve the Standing Long Jump Performance? A Mininarrative Review

**DOI:** 10.1155/2020/8829036

**Published:** 2020-12-17

**Authors:** Huiyu Zhou, Peimin Yu, Anand Thirupathi, Minjun Liang

**Affiliations:** ^1^Faculty of Sports Science, Ningbo University, Ningbo, China; ^2^Research Academy of Grand Health, Ningbo University, Ningbo, China

## Abstract

Standing long jump (SLJ) is complicated by the challenge of motor coordination in both the upper and lower segments. This movement is also considered to be a fundamental skill in a variety of sports. In particular, SLJ is an important test index for middle school students for assessing their physical fitness levels. This assessment takes the form of a physical fitness test high school entrance examination in some countries such as China. This minireview summarizes recent studies that have investigated how to improve the standing long jump performance from different aspects which include arm motion, takeoff angle, standing posture, warming-up exercise, and handheld weight. The common study limitations, controversial knowledge, and future research direction are also discussed in detail.

## 1. Introduction

Jumping is a fundamental movement skill in a variety of sports that needs the complex motor coordination of upper and lower limbs to obtain a good performance, such as volleyball, basketball, ski jumping, and some ball sports in which the high velocity of muscle contractions is required. Standing long jump (SLJ) is considered a good predictor of sprint and jump performance, which presents correlations highly with isokinetic measures of lower extremity force [1].

The SLJ is an important physical fitness test index for middle school students in China. This assessment metric takes the form of a physical fitness test high school entrance examination in China. More often than not the outcome of this physical fitness test determines the eligibility of the student to be admitted to their high school of choice. Therefore, the SLJ score is of particular importance, and examining methods to effectively improve SLJ performance could be beneficial to middle school students. Previous researchers have also investigated various aspects of the SLJ ([2–4]. These studies have investigated body configuration and joint function of both upper and lower segments between adults and preschool-age children [3] and explored the significant correlations between a variety of isometric, kinetic, kinematic, and SLJ performance parameters [2, 4]. The category of jumps can be divided according to the arm motion. i.e., jumps with restricted arm motion (JRA) and jumps with free arm movement (JFA). In terms of comparing the JRA and JFA jump categories, the influence of arm movement on SLJ performance was explored with respect to understanding whether the jumping distance could be increased by arm swing [5]. To detect more biomechanical mechanisms for improving the movement performance, the optimum takeoff (TO) angle 29°-38° of SLJ in adult males was found, although the biomechanical evidence for this result is unclear [2, 3, 5]. Meanwhile, the different TO positions for SLJ have also been studied by Mackala and associates where the different results of parallel or straddle foot starting placement for the quality of SLJ were determined [6]. Moreover, Koch et al. explored the potential effects of stretching and warm-up activities on the SLJ in moderate and well-trained subjects. The results presented show that warm-up activities had a slight effect on jumping performance, while maximum muscles strength showed a significant correlation with jumping ability [7]. On the other hand, according to the research by Minetti and Ardigo, the hand with halteres increased the TO speed in the SLJ mainly because the muscle exerted more force in the moderately loaded subjects in comparison to the nonloaded scenario [8]. The researchers compared the effects of hand-holding different weights on the kinematic and dynamic characteristics of SLJ subjects, and the relationship between the hand-held weight and jumping performance was clarified (Fukashiro et al. 2005; [8]).

Besides, the biomechanical characteristics of SLJ from a computer modeling perspective have been investigated by Hickox et al. Hickox and colleagues verified the effectiveness of SLJ modeling based on the two-dimensional sagittal plane evaluation, and the results showed that plane analysis was sufficient to detect lower limb movement [9]. In addition, Ashby and Delp documented that arm activity can improve the SLJ performance by using the optimal control simulation method [10]. These have provided us with an insightful understanding of the sports coordination mechanism of SLJ.

To date, a narrative review on the effect of motor activity on the standing long jump performance remains unavailable in the literature. Therefore, the purpose of this article was to summarize the methods for coaches and trainers to improve the SLJ performance from the perspective of several aspects based on previous studies.

## 2. The Different Analytical Aspects of the Standing Long Jump

### 2.1. The Role of Arm Motion in the Standing Long Jump

Many previous studies have elucidated the role of arm movements in various jump activities [11]. There are several benefits to arm motion, such as arm swing increases the velocity of the body's center of gravity (CG) at TO, acquires the larger peak magnitude of the vertical ground reaction force, and creates an additional downward force on the body which allows for greater muscle force development [11–13]. To be more specific, Ashby and Heegaard have revealed the biomechanical mechanism of the role of an arm in the SLJ [5]. They conducted a comparative study between JFA and JRA subjects; the results showed that the average distance improved by 21.2% in the JFA group compared to JRA, the average velocity of the CG increased by 12.7% at TO, and the horizontal displacement of CG before TO significantly increased among the JFA subjects when compared to JRA subjects. In terms of kinetics, the peak value of horizontal ground reaction force (HGRF) in the JFA group was also significantly increased when compared to the JRA group. Additionally, it was considered that majority of the improvements observed in the SLJ were attributed to the increased CG velocity at TO during arm movements.

Three different theories have been proposed to explain the principle of how CG velocity was increased by arm movement at TO. The theory of “hold back” indicated that the lower limb extensor was activated by arm motion during the propulsive phase to limit excessive forward rotation, which would achieve an optimal landing. On the contrary, if arm motion was restricted, the jumper must “hole back” to limit the lower limb extensor thereby avoiding excessive forward rotation of the trunk and legs that would limit proper landing [5]. The theory of “joint torque augmentation” suggests that the arm swing creates a downward force on the shoulder, which slows down the shortening velocities of the lower extremity joint extensors thus resulting in a greater muscle torque [11, 12]. The “energy transfer” theory is that muscles in the shoulder and elbow joints transfer energy to the rest of the body before takeoff, increasing the speed and displacement of the CG in both horizontal and vertical directions [12]. Ashby assessed the reliability of all three theories in jumping movement by using the optimal control simulations; it was found that the “energy transfer” theory is the primary mechanism for increasing the velocity of the CG in JFA at TO, because the large work of the upper limb joint muscles is produced by free arm movement which can be effectively transferred to the lower limb [14]. Above all, jumping with a free arm movement can significantly improve SLJ performance.

### 2.2. The Optimum Takeoff Angle of CG

The trajectory of CG movement can be likened to a projectile in the flying phase of the SLJ. Therefore, an appropriate projection angle is identified as a crucial factor to develop an ideal performance. Previous studies have suggested that the projection angle between 29° and 38° has been considered as an optimum TO angle for jumpers, but the biomechanical reasons for this projection angle option are not well explained [2, 3, 5]. However, the results showed that the TO angle was not the main factor contributing to a successful SLJ performance, especially that the distance affecting by TO speed was more important than TO angle [15]. In order to obtain maximum TO speed, the optimum TO angle in SLJ was suggested to be less than 45° [15]. Additionally, the authors also suggested that spiked shoes should be used at very low takeoff angles to increase traction at TO phase so as to reach a greater jump distance. There are few researches that have been done on the optimum takeoff angle in SLJ movement. Further studies should be conducted in the future to verify the role of appropriate TO angle in SLJ.

### 2.3. The Standing Posture of SLJ

The coordination strategies of a jumper can be affected by different standing postures. Despite the conclusions by previous researches suggesting that jump distance is insensitive to the initial position, which is determined by angle of knee flexion and posterior angle of the trunk at TO phase, the initial postures play an important role in SLJ movement for attaining a good performance [16]. Actually, the effects of various foot positions on the quality of SLJ have been studied extensively specifically from parallel and straddle position perspectives. The parallel SLJ setup involves placement of the feet at shoulder width apart or more and parallel to the starting line. The straddle SLJ setup contrastingly involves placement of the feet in self-selected straddle position ranging from 30 cm to 40 cm with one of the feet in front. Mackala and colleagues have investigated the effect of the differences in kinematics and kinetics between parallel and straddle placement in SLJ movement. In their study, three related muscle group activities were evaluated by electromyography (EMG) in different foot placement groups. The results showed that the average distance can be improved by 5.18% in the straddle position when compared to the parallel position. More specifically, larger flexion angles at the trunk, hip, and knee joints were observed in the straddle position. Larger peak joint moments were also found at straddle feet placement in comparison to the parallel position. The subject's whole body was more likely to tilt forward in the straddle position and produce a lower center of mass that can generate a larger momentum in the forward and upward movements, thus contributing to a better performance. In contrast to parallel posture, the greatest muscle activation was observed in the gluteus maximus and biceps femoris during the push-off phase in the straddle starting foot position, and the lower limb extensor muscles such as gluteus maximus and biceps femoris could exert more force in the straddle position compared to parallel position [6].

Besides the experimental measurement of SLJ, long jump simulation researches have also been conducted. The numerical simulation could take the advantage of decreasing the biased effects. In order to effectively study the influence of starting posture on SLJ, a planar 4-segment human model has been established by Cheng and Chen [18] to detect the joint torque activation level and TO time in SLJ movement. Three different starting postures included the squat, low squat, and high squat were tested; the height of the squat was determined by the initial center of mass heights at 78 cm, 88.4 cm, and 62.9 cm, respectively. However, the results showed that the jump distance was slightly dependent on the initial posture [18]. It is a little difficult to draw a conclusion based on the current researches regarding whether SLJ performances can be influenced by starting posture, since different strategies of starting posture in selected articles have been used. One of the articles focused on the feet placement [19], and another was concerned about the height of squat [20]. We may be able to get some information from limited studies including preliminary studies to provide clarity in understanding the effects the straddle starting feet placement may have on jump distance during the SLJ movement. To fully understand the complexities associated with improving performance in the SLJ, further investigations into feet placement, different squatting heights, and other postures associated with the SLJ need to be investigated and understood so that future projects can provide more valuable information to the jumper and coaches.

### 2.4. The Effect of Warm-Up on the SLJ

The warm-up exercises are considered as an important factor for injury prevention and a prerequisite for good athletic performance. Stretching movements have been widely applied in warm-up exercises for training and competition purposes in a variety of sports [7]. Researchers have shown that after warming up, the muscle's stiffness is reduced and relevant muscles have more compliance before the sporting activity is started [21]. Furthermore, some studies have found that stretching contributes to a negative effect on muscle strength, performance, and strength endurance. [22–25]. Similarly, Koch et al. also detected the negative effect of different warm-up exercises which included stretching, high force, and high power in trained and untrained men and women. According to this research, the results revealed that no significant differences were found in any warm-up exercise routines [7]. It was demonstrated that the effect of warm-up exercises on SLJ performance was not obvious, and the muscle strength was strongly associated with jump ability. This finding is consistent with the conclusion drawn by Koch and colleagues who found that no effect on sports performance was observed during their investigation of a static stretch involving a standing/seated toe touch and standing/seated quadriceps stretch [7]. Even in the vertical jump movement, previous researches have indicated that a small (3%) reduction in height of the vertical jump was found after the performance of proprioceptive neuromuscular facilitation stretching [8]. Above all, the adverse effects of warm-up exercises on SLJ sports performance have been consistently confirmed by previous researches; therefore, the warm-up exercises are not recommended for SLJ movement.

### 2.5. The Function of Handheld Weight on SLJ Performance

The effect of handheld weights on jumping performance has been conducted by a few studies [8, 26]. Papadopoulos and associates demonstrated that each hand carrying a 3 kg load would contribute to a 6% increment in the jump distance performed at the same TO speed. In addition, the computer simulation presented when subjects were jumping with 2 kg to 9 kg weights in each hand showed that the velocity of TO can be increased by 5-7% [27]. The loading effect during jumping allowed muscles to exert larger strength which led to a reasonable muscle contraction [27]. Researchers have compared the different effects of various handheld masses on the kinematic and dynamic features of SLJ [8]. They suggested that better SLJ performance could be achievable with extra weights between 3 kg and 6 kg due to the larger horizontal translation of the COM and the greater GRF that was yielded. This conclusion is consistent with Lenoir and associates who showed that a jump distance of 13.88 ± 0.70 cm was achieved without loads while the distance was significantly increased with extra weights (14.64 ± 0.76 cm) [28]. Ashby also indicated that jumpers who carried a 4.6 kg loading increased their jump distance by 0.39 cm [26]. Furthermore, using a simulation analysis, Minetti and Ardigo noted that a 5 kg to 6 kg load is the optimal weight for increasing jump distance [27]. Subsequently, Huang et al. tested the optimal weights for SLJ jumpers and found it to be 5.6 kg (Huang et al. 2005). According to the analysis presented, the improvement in SLJ performance by extra weight is mainly attributed to greater GRF force and greater takeoff velocity of COM in the horizontal direction. Therefore, the method of holding extra loading to improve SLJ performance can be applied in a training program for different sports purposes.

## 3. Conclusion

Many studies reveal the effect of the object on standing long jump from a different perspective. The five methods that could influence the SLJ performance were included in this mininarrative review, in which the arm motion, takeoff angle less than 45°, and 5 kg-6 kg handled weight play a positive effect on SLJ performance. All these biomechanical variables identified as the main factors to achieve an ideal SLJ performance generally improved takeoff velocity of COM and increased the power of the lower extremity. On the other hand, warm-up exercises have presented a negative influence on SLJ movement since it reduces the muscle's stiffness and increases muscular compliance. There was a contradictory view in the starting posture of SLJ movement as indicated by the different strategies of starting posture in selected articles. Further studies on muscle activities in the lower extremities during the SLJ movement are needed since muscle strength is a determining factor to achieve better performance. On the other hand, the application of specialist jumping shoes in SLJ movement is also an important research topic since running shoes have been extensively investigated; however, to date, no research has focused on jumping shoes.

## Data Availability

The data that support the findings of this study are available from the corresponding author upon reasonable request.
